# Multimedia Character Modeling Design and Modeling of Cartoon Animation Based on Bayesian Sequence Recommendation Algorithm

**DOI:** 10.1155/2022/9205227

**Published:** 2022-01-10

**Authors:** Hao Wu, Shi-Jiang Wen, Jong-Hoon Yang

**Affiliations:** ^1^Department of Digital Image in Sangmyung University, Seoul 03015, Republic of Korea; ^2^School of Animation and Digital Arts, Communication University of Zhejiang, Hangzhou 310018, China; ^3^Department of Xinjiang Art and Sports, Ningbo Childhood Education College, Ningbo 315016, China

## Abstract

With the continuous development of the social economy, cartoon animation and other multimedia and streaming media forms are becoming more and more popular and are loved by all kinds of people, such as monkey king and Nezha. However, the multimedia of these cartoon animation needs to conform to mainstream values and transmit positive energy. In view of these needs and shortcomings, this study relies on the Bayesian sequence recommendation algorithm, combs the three-tier architecture diagram of multimedia character modeling, analyzes it, respectively, from the perspectives of hierarchy, behavior, and interactive process, and tries to build corresponding animation design management documents, so as to provide corresponding decision-making basis to produce animation and develop corresponding results, provide corresponding reference mode for cartoon animation multimedia character manufacturing, complete corresponding cartoon animation multimedia characters faster, and improve cartoon animation multimedia works and efficiency. The simulation results show that the Bayesian sequence recommendation algorithm is effective and can support the design and modeling of cartoon animation multimedia characters.

## 1. Introduction

With the continuous development of the social economy, cartoon animation and other streaming media continue to be popular all over the world, especially the continuous integration of culture, the original cultural barriers are gradually eliminated, and the Eastern and Western cultures have become the embodiment of many artistic values [1, 2]. Especially for the characterization of cartoon characters, such as the Oriental Monkey King, Nezha, and other emerging characters, they occupy an important position in the whole animation and other cultures and are very popular with all kinds of people [3, 4]. Different visual symbols are not only the needs and constituent elements of animation action but also the basic form of esthetic art development, which is also one of the necessities of many life decorations and artistic modeling [5, 6]. The image inpainting technology based on variational partial differential equations reconstructs the image model. A new function is formed by combining the L2 energy of image gradient and total variation, and it is introduced into the optimization problem. The dynamic behavior of the model is formed through the threshold function, and TV items are applied in high-density areas to retain the most important image features. The threshold function is an evolutionary partial differential equation with asymptotic control, which is more suitable for complex images [7]. Based on the multisink distributed power control algorithm suitable for coal mine roadway, the multisink network is combined with the clustering Voronoi scope routing algorithm by using the multisink network structure and the idea of nonuniform clustering. It assigns the best transmission range and power to each receiver, uses each receiver as the cluster head, and performs network clustering. On the basis of ensuring good network coverage, the network topology is optimized [8].

In the process of the ancient art design, people's worship of celestial bodies tends to more understand the circle, which is not only the beginning of the history of the circle but also people's understanding of the circle. Therefore, the shape of the circle is everywhere in various design processes in the world. In the actual modern process, the circle is also an essential element, such as a circular camera, circular bus card, and circular coin. The consciousness of “round sky and place” can also be seen everywhere in life, which is also the popularization and development of circular elements. The simple simplification, multichange, perfection, resonance, and other characteristics can be accepted by everyone, and new laws can be found from these morphological laws, such as the design of the temple of heaven and the temple of the earth [9, 10]. It is precisely because these simple elements, such as squares and circles, gradually form complex cartoon images, so as to realize the design of visual elements in different animation character modeling design, such as the character's face, eyes, and other parts [9, 10].

Circular modeling has a certain reduction in the modeling design of animation characters, and people gradually restore the corresponding animation modeling effect from this form [11, 12]. In the process of animation modeling, the first thing to be solved is the style related to art. Only after the style is determined, the remaining work can be implemented step by step and the corresponding tone of the whole film is determined [13, 14].

In view of these limitations and needs, based on the Bayesian sequence recommendation algorithm, this study combs the corresponding architecture modeling of cartoon animation multimedia robbery, analyzes the corresponding art style, creates the role conception method with the corresponding architecture description language, and uses the corresponding ruler for action analysis so that the corresponding modeling can better fit the previous role, so as to improve the corresponding animation design efficiency, shorten the corresponding production cycle, and improve the design effect and quality.

## 2. Present Situation of Animation Multimedia Character Modeling

For multimedia cartoon characters, their biggest engineer is a complex and huge systematic project, which requires human, material, time, and other inputs to be comprehensively completed, rather than transient and temporary performance. Whether it is character modeling or 3D animation, its production is a very complex process, as shown in Figure 1, and the corresponding process involved is shown in Figure 2.

Excellent animation work is inseparable from an excellent script. When the corresponding ideas of the screenwriter are transformed into the corresponding excellent script, the complex text script can be transformed into complex animation films, especially complex animation films with different cultures [15, 16]. This is not only a complex design and screenwriting process but also a very challenging work, which requires advanced planning and corresponding pre-mid-production and postproduction. In the early stage, the production of written scripts is extremely important.

Animation scripts come from a wide range of sources. They can be written according to the corresponding idea or a proverb, or from myth or prose, but in any case, they need to be converted into corresponding text scripts.

Animation scripts have a wide range of origins. They can be compiled based on a proverb, or they can be compiled from ancient myths or prose novels. Regardless of the source, they need to be compiled into scripts that can be easily transformed into pictures.

A little monk hurried up the mountain.

One inadvertently fell and sat up and saw that he was stepping on the back of a big tortoise. The tortoise turned over and couldn't crawl. The little monk turned it over and let it crawl away.

There is a small temple on the high mountain.

There is a Guanyin Bodhisattva in the temple, holding a clean bottle with willow branches inserted in the bottle.

The young monk went to the temple and worshipped Guanyin Bodhisattva first. He saw the willow branches hanging down in the clean bottle. He took the clean bottle and poured it. There was not a drop of water in the bottle.

The little monk picked up the bucket and pole, and went down the mountain to carry water.

He worked hard to pick up two buckets of water and came to the mountain, first filled the water tank, then filled the net bottle, and then sat down to do his homework—knocking on the wooden fish to recite sutras.

The sun came out from the eastern hills and set down on the western hills, passing like this day by day.

The little monk chanted every day. Once he bowed his head and opened his eyes to see that a mouse was looking at him by his head. The little monk raised the gavel and knocked it head on at the mouse. The mouse ran away in fright. The little monk laughed.

Through the storyline in the script to present the personality characteristics of the character, there is a common problem in this: the director and the stylist will have different definitions of the character image after reading the text script, and how does the styling designer follow the text script and more completely and quickly understand the director's concept, reduce deviations, and finally complete the character modeling renderings. This is the first problem to be solved in the preproduction process of animation. The cultural and professional qualities of the director and the animation designer determine this, namely, the size of the deviation. An excellent animation director can control the size of the deviation through profound cultural cultivation and profound knowledge, and an excellent styling designer can understand the director's design of the script while absorbing text scripts through strong cultural literacy and professional skills, such as ideas, recreation, and completion of the final design. This study will use the SBC architecture description language to build and manage the character modeling design in the animation art modeling style. The use of animation character design management documents can solve the problems from the text script to the modeling style of the whole film, realize the image requirements of directors and stylists, and provide reference for the preproduction of other character animation short films, so as to shorten the time of preproduction artistic style and improve the production efficiency.

In order to cooperate with the project production and management of animation films, the structure and behavior integration structure-oriented character animation short film art style character design management file is constructed, and the character design structure and behavior in the character animation short film art style are clearly expressed. The interactive relationship has 4 purposes:

1. Through the use of the SBC system architecture description language, the structure and behavior of the character design in the production process of the art modeling style of the animation preproduction are explored, and the character modeling design model of the architecture-oriented animation preproduction art style is established.
2. The architecture-oriented and nonarchitecture-oriented models are evaluated, and the best character design model is proposed as a system file for animation character design management. The purpose is to improve the current character designer's inability to absorb the text script while comprehending the director's design ideas, so as to carry out a recreative design of precise creation and to improve this deficiency through the design of the management file.
3. The character design creation method is improved in the art modeling style of the current animation preproduction, and its management files are designed through the SBC system architecture description language so that the stylist can quickly grasp the director's design ideas and establish the art modeling style design of the entire short film and the overall picture, enhance the understanding of the stylist's script, and enhance their business ability and the quality of the design of the work.
4. The results of this project can be used in the character modeling design in the preproduction art modeling style of other animated short films of the character category, as the basis of its reference.

## 3. Bayesian Sequence Recommendation Algorithm

### 3.1. Cross-Use SBC System Architecture in Multiple Fields

This study uses the corresponding system architecture to describe the animation language, expounds the corresponding animation for different animation languages, specifies the corresponding animation style, role design structure view, and behavioral view, and constructs the corresponding role design management model. At present, the preproduction of animation is based on text scripts, but there is generally no clear language description of the modeling style in the text scripts. Therefore, communication between the director and the stylist is not allowed during the animation production process. To avoid cognitive deviations, using the SBC architecture description language in System Science 2.0 to present the role images of the director and stylist in the text script in the form of an architecture-oriented role design management file can make up for the deficiencies in this process.

#### 3.1.1. Summary of Role Design Management Documents for Animation Art Style Modeling

For animation character art style for role design in modeling, animation directors can use the corresponding animation reference documents for animation production and key supervision of each link.

For different architectures, we can analyze the corresponding information loss of animation production so that the later production personnel can more clearly understand and grasp the early director's design ideas, use the animation role design management documents, more clearly find the director's design of animation role modeling, and analyze the corresponding style of modeling. Similarly, according to the corresponding character relationship, we can get a series of animation pictures.

For character design, the style balcony can be analyzed and reshaped according to the requirements of the animation director. The animation director can let all animation producers understand their ideas and logic according to the corresponding design principles and design ideas, so as to realize the sharing of information and docking of ideas in the production process [17, 18].

#### 3.1.2. Role Design Management Rules

*(1) Advantages of Using SBC Architecture Method to Build Role Design Management*. For the role design management of art modeling style, it is very important. The role design management not only needs to filter the impossible part of the work but also needs to deal with the director for design. Only in this way we can solve the communication between directors and stylists, improve work efficiency, shorten the work cycle, and save corresponding production costs.

*(2) Role Design Management File Construction in Animation Art Modeling Style*. The corresponding animation modeling management rules and methods are researched and used, the script through the corresponding documents is sampled and analyzed, the framework is clearly defined, and the specific integration requirements are clarified [19, 20].

### 3.2. Construction and Decomposition of Sequence Transfer Tensor

Let *U*={*u*_1_, *u*_2_,…, *u*_*M*_} be the user set and *I*={*i*_1_, *i*_2_,…, *i*_*N*_} be the commodity set. The calculation of the animation probability of the user from the current browsing at time *t* is shown as follows:

(1) $$\begin{array}{c} x_{u,i,j}=p\left(i\in I_{u}^{t}|I_{u}^{t-1}\right). \end{array}$$

The recovery calculation of each element in the tensor can be expressed as follows:

(2) $$\begin{array}{c} x_{u,i,j}^{\prime }=v_{u}^{U,K},v_{j}^{K,U}+v_{J}^{K,I}\cdot v_{i}^{I,K}+v_{u}^{U,I}\cdot v_{i}^{I,U}, \end{array}$$

wherein *v*_*u*_^*U*,*K*^ and *v*_*j*_^*K*,*U*^, respectively, represent the latent vectors of the user and the next commodity. Since *v*_*u*_^*U*,*I*^ and *v*_*i*_^*I*,*U*^ are independent of the next commodity *J* to be predicted and do not affect the final sorting result, a more concise expression is obtained as follows:

(3) $$\begin{array}{c} x_{u,i,j}^{\prime }=v_{u}^{U,K}\cdot v_{j}^{K,U}+v_{j}^{K,I}\cdot v_{i}^{I,K}. \end{array}$$

The problem is converted into a list sorting problem, as shown in the following formula:

(4) $$\begin{array}{c} j^{\left(1\right)}{>}_{u,i}\cdots {>}_{u,i}j^{\left(k\right)}\Leftrightarrow {\hat{x}}_{u,i,j\left(1\right)}>\cdots >{\hat{x}}_{u,i,j\left(k\right)}, \end{array}$$

where *j*^(*k*)^ represents the position of goods in the list and ${\hat{x}}_{u,i,j\left(1\right)}$ represents the transfer score of users *u* from goods to goods.

### 3.3. Bayesian Sequence Optimization Algorithm

In this study, the Bayesian optimization algorithm based on the list is used for parameter optimization. The specific maximum a posteriori probability is shown as follows:

(5) $$\begin{array}{c} p\left(\Theta |{\text{list}}_{u,i,j}\right)\propto p\left({\text{list}}_{u,i,j}|\Theta \right)p\left(\Theta \right). \end{array}$$

The maximum a posteriori estimation method is used to estimate the model parameters, as shown in the following formula:

(6) $$\begin{array}{c} \arg\max_{\Theta }\prod_{list_{u,i,j}\in D_{x}}p\left({\text{list}}_{u,i,j}|\Theta \right)p\left(\Theta \right). \end{array}$$

The maximum a posteriori probability estimation of personalized sorting is shown in the following formula:

(7) $$\begin{array}{c} \arg\max_{\Theta }\prod_{list_{u,i,j}\in D_{x}}\ln\left(p\left({\text{list}}_{u,i,j}|\Theta \right)\right)-\frac{\lambda_{\Theta }}{2}{\left\|\Theta \right\|}^{2}+C. \end{array}$$

The likelihood function can be calculated by

(8) $$\begin{array}{c} p\left({\text{list}}_{u,i,j}|\Theta \right)=\prod_{m=1}^{k}\frac{\phi \left({\hat{x}}_{u,i,j\left(n\right)}\right)}{\sum_{n=m}^{k}\phi \left({\hat{x}}_{u,i,j\left(n\right)}\right)}, \end{array}$$

where *k* represents the length of the list and the activation function. *ϕ*(·) defines *ϕ*(·) as an exponential function. By integrating formula (8), the change in the objective function is shown as follows:

(9) $$\begin{array}{c} \arg\max_{\Theta }\sum_{list_{u,i,j}\in D_{x}}\sum_{m=1}^{k}\left\{{\hat{x}}_{u,i,j\left(m\right)}-\ln\sum_{n=m}^{k}\exp\left({\hat{x}}_{u,i,j\left(n\right)}\right)\right\}-\frac{\lambda_{\Theta }}{2}{\left\|\Theta \right\|}^{2}. \end{array}$$

The map descent method is used to optimize formula (9), and the parameter update expression is obtained as follows:

(10) $$\begin{array}{c} \Theta^{\prime }=\Theta +\alpha \left(\frac{\partial }{\partial_{e}}\left(\ln\left(p\left({\text{list}}_{u,i,j}|\Theta \right)\right)-\frac{\lambda_{\Theta }}{2}{\left\|\Theta \right\|}^{2}\right)\right), \end{array}$$

where *α* > 0 indicates the learning rate.

## 4. Simulation Experiment

The simulation experiment is designed from multiple perspectives, mainly including structural and behavioral design (Figure 3), using the corresponding three-tier frame diagram for the corresponding animation form design, specifically defining and making the animation shape, and using the structure form diagram for animation interpretation and management (Figure 4). The style of animation art modeling, role design, and corresponding action interaction is expressed through the interactive flowchart, as shown in Figure 5.

1. SBC architecture form: a system includes structural viewpoints, behavioral viewpoints, and other viewpoints. Among them, structural viewpoints and behavioral viewpoints are the two most important viewpoints of the system. The SBC architecture is to comply with the requirements of the unification of structure and behavior. Through its integrated architectural model, all views are described and expressed at the same time. When used in the character design of animation production, the biggest advantage is that no matter how complex the animation script is, it can enable the director to communicate better with the stylist, clearly and efficiently present the definition of the role design of the film, and avoid the loss of information in the communication process. It can be seen that the integrated approach of the SBC architecture can not only run in different professional fields but also be applied to different fields of the same professional.
2. SBC architecture description language construction of the animation character design system model: when the stylist designs the art style at the early stage of animation, he will first take the design of the character as the main style. Because the creative personnel are restricted by their own cultural accomplishment and professional quality, the character modeling he designs and draws is habitually partly subjective color. After communicating with other people in the animation production, especially after understanding the director's intentions, some new ideas will be generated. Usually, a stylist has two steps when designing at this stage: first, he creates according to his own conception of the character modeling in the script, that is, he must be familiar with the script and understand the plot when he gets the first-hand information for the modeling task. To study the script, the main information of the characters in the play must be grasped, and some element information related to the modeling in the play must be found. Sometimes the fate of the characters in the script and the development of the story plot also hint at the information related to the modeling. That is, the stylist needs to be familiar with the script before drawing the sketch, and the sketch should be as concise as possible to make it easier to highlight the effect. Then, the design sketch is submitted to other animation production staff for study and discussion and then is reviewed by the director, expressing his views on the styling. After the director has expressed his own ideas, the stylist will proceed according to the director's explanation and integrate other useful information. Reprocessing can also be said to be recreation. When recreating, the focus is to correct the lack of understanding of the role information in the play and to maximize the strengths and avoid the weaknesses.

The characters in cartoons are just like actors in movies. How to choose actors to play the story is like designing what kind of characters to express the story. The character design in animation creation is as important as the selection of actors in a movie. What kind of image the character looks like, whether it is fat or thin, whether it is young or old, whether it is the protagonist or supporting role, etc., are all factors to be considered when creating. When designing a character in an animated short film, a stylist uses the script as the basis. Under normal circumstances, he will think about the main components of the character design, the character's personality information, background information, visual information about the character, and so on.

From the interactive design flowchart of animation roles, it can be seen that the animation design interacts with the designer and finally submits for review and exchange to realize information feedback, make the personnel in the animation production process more clearly understand the whole animation design style and ideas, delegate more choices to the later animation production personnel, and give full play to their advantages and imagination, so as to quickly and well complete the role design of animation short films (Figure 5).

The psychological basis of animation modeling is human recognition of images, colors, and other modeling. The closer the corresponding modeling design is to the essence, the more it can become a classic. In particular, the shape shaping and character analysis of characters often contain their internal essence and subconsciously help and promote the development of stories, especially for animation characters. The modeling of its animation characters should have distinct characteristics and be extremely significant, such as car stories and other animation films can be clearly seen.

In the process of character creation, character modeling often uses multiple elements, such as circles and squares. However, with the continuous development of technology, especially the development of three-dimensional technology, a variety of shapes are further hybrid, and the production efficiency and cost are changed. The modeling of animation characters no longer only pursues complex design but prefers to use color, shape, and other aspects of design. On the one hand, the design of animation modeling characters returns to the initial starting point.

### 4.1. Role Design Architecture Form Management Document

For the modeling animation design, we first need to use the role management design to design and analyze the corresponding architecture hierarchy diagram, as shown in Figure 6. Taking an animation short film as an example, we can uniformly integrate the relevant information such as the type, appearance, number, main and secondary characteristics, and style of the role and describe it in the form of pictures and texts.

The specific process of role interaction is described in Figure 7. From the results of Figure 7, we can see the communication results between the relevant directors of modeling and the later animation designers for the female main animation modeling of the short film, which are redescribed in the form of pictures and words. After being jointly confirmed by both parties, the later animation designers give full play to and create according to this result and present corresponding effects, expressions, and thematic maps so that other later stylists can also create corresponding roles and unify style and color.

### 4.2. Comparing Nonarchitecture- and Architecture-Oriented Approaches

At present, in the early stage of the current animation production market, the communication between animation directors and corresponding stylists is only limited to oral communication and personal understanding, which will lead to errors in information transmission and the first floor. If you simply interpret all modeling information with personal subjectivity, you cannot recognize it through the overall concept. At the same time, it is impossible to understand the modeling design ideas of the animation director, which may lead to the deviation between the actual creative effect and the director's idea.

The Bayesian sequence recommendation algorithm proposed in this study is compared with the corresponding traditional algorithm. The experimental results are shown in Figures 8 and 9. With the increase in the number of animation modeling recommendations, the corresponding recommendation accuracy shows a decreasing trend, and the recommended recall shows an upward trend. From the simulation results, the Bayesian sequence recommendation algorithm (BSRA) is superior to the traditional methods and has the corresponding improvement over MTF and BPR algorithms. At the same time, it also alleviates the sparsity of animation modeling data to a certain extent.

In order to verify that the algorithm in this study can effectively solve the problem of data sparsity, further experimental analysis is carried out on training datasets with different densities. The experimental results are shown in Figure 9. The experimental results show that the error of the MF algorithm is the largest, followed by PMF, which analyzes the user behavior transfer. The three-dimensional tensor must be transformed into a user order algorithm. This is because MF and PMF algorithms can only act on the two-dimensional matrix as column transfer pairs, which will lead to the loss of user behavior transfer relationship. TF algorithm based on three-dimensional tensor is much higher than MF and PMF algorithms. This is because the TF algorithm can capture the internal relationship of animation modeling. The RMSE error of the BSRA algorithm proposed in this study is much smaller than the traditional matrix decomposition algorithm. On the dataset with a density of 50%, the error rate of the BSRA algorithm significantly decreases, and the RMSE decreases with the increase in data density. This is because the algorithm proposed in this study makes full use of observed data and unobserved data. The simulation results show that the Bayesian sequence recommendation algorithm is effective.

## 5. Conclusions

With the continuous development of the social economy, cartoon animation multimedia character modeling is loved and favored by all kinds of people, but for the animation modeling design of the east and the west, how to seamlessly convey the design concept is extremely important. Based on the Bayesian sequence recommendation algorithm, this study manages and designs the corresponding cartoon animation multimedia role modeling and uses the role design ideas to show which can further improve the design ideas of animation modeling, share the direction and style of animation directors, and all relevant stakeholders in postproduction can directly and clearly understand the ideas. It avoids unnecessary barriers to information sharing, effectively reduces the traditional communication cost, and improves the design idea and efficiency. The simulation results show that the Bayesian sequence recommendation algorithm is effective, can support the modeling design and modeling of cartoon multimedia characters, and can produce competitive animation multimedia films.

## Figures and Tables

**Figure 1:** Flowchart of traditional and digital animation production.

**Figure 2:** Flowchart of 3D animation production.

**Figure 3:** Role design architecture hierarchy.

**Figure 4:** Integration of role design structure and behavior.

**Figure 5:** Interactive flowchart of role design.

**Figure 6:** Hierarchy of character design in Miyan.

**Figure 7:** Interactive flowchart of character design in Miyan.

**Figure 8:** Variation of accuracy with recommended quantity.

**Figure 9:** Change in recall rate with recommended quantity.

## Data Availability

The labeled dataset used to support the findings of this study is available from the corresponding author upon request.
